This article has been retracted.

# Efficacy of Xiyanping in the Treatment of Elderly Patients with Chronic Obstructive Pulmonary Disease and Its Effect on the Expression of GDF-15 and HIF-1*α* in Serum

**DOI:** 10.1155/2022/6193110

**Published:** 2022-10-12

**Authors:** Jun Xia Wang, Ying Zhang, Shu Fang Wang, Juan Li, Peng Cheng Li

**Affiliations:** ^1^Pharmacy Department of Shijiazhuang Eighth Hospital, China; ^2^Department of Anesthesiology, Shijiazhuang Eighth Hospital, China; ^3^Department of Internal Medicine of Tang County Hospital of Traditional Chinese Medicine, China; ^4^Department of Internal Medicine, Langfang Hospital of Traditional Chinese Medicine, China

## Abstract

**Background:**

COPD is a chronic respiratory disease with a long course and recurrent characteristics. According to relevant statistics, the global incidence of COPD is more than 30%, which seriously affects the life of patients and endangers their health.

**Objective:**

To observe the curative effect of Xiyanping in elderly patients with COPD and its influence on the expressions of growth differentiation GDF-15 and HIF-1*α* in serum.

**Methods:**

From August 2019 to December 2021, 86 elderly patients with acute exacerbation of COPD were admitted to our hospital. As the research objects, they were divided into the control group (*n* = 43) and the observation group (*n* = 43) randomly. The control group received the conventional treatment, while the observation group got Xiyanping on the basis of the control group. The differences in the duration of antibiotic use, expectoration, hospital stays, adverse reactions and serum-related factors, blood routine, pulmonary function, airway hyperreactivity index, COPD assessment test (CAT) score, and Borg score were made a comparison between them.

**Results:**

On the 3rd and 7th days after being treated, the sputum excretion in them was higher than before, but on the 3rd day of treatment, the sputum excretion in the observation group was higher than that in the control group, while on the 7th day of treatment, the sputum excretion was lower than that in the control group with statistically significant differences (*P* < 0.05). Before treatment, the serum-related factors and blood routine indexes between them were similar (*P* > 0.05). After treatment, GDF-15, HIF-1*α*, CXCL12, TNF-*α*, IL-8, TGF-*β*, WBC, and NEU in them were significantly lower than before, and the values in the observation group were significantly lower than those in the control group with statistically significant differences (*P* < 0.05). There was no difference in the related indexes of pulmonary function and airway hyperreactivity between them before treatment. After being treated, FEV1, FVC, and FEV1/FVC in them were significantly higher than those before treatment. The airway resistance and lung compliance of the two groups at exhalation and inspiration were significantly lower than before, and the values in the observation group were significantly lower than those in the control group (*P* < 0.05). There was no difference in CAT and Borg scores between them before treatment. After treatment, the CAT score and Borg score of these patients were significantly lower than those before treatment, and the value of the observation group was significantly lower than that of the control group (*P* < 0.05). The duration of antibiotic use and length of stay in the observation group were significantly shorter than those of the control group, while the incidence of adverse reactions was not statistically significantly different compared with the control group (*P* > 0.05).

**Conclusion:**

Xiyanping can improve pulmonary function of elderly patients with acute exacerbation of COPD, reduce the response of airway hyperreactivity, and promote the excretion of sputum.

## 1. Introduction

Chronic obstructive pulmonary disease (COPD) in the elderly is a common clinical respiratory disease, featured by incompletely reversible airflow limitation, and the disease develops in a progressive way [1]. As a risk factor for acute exacerbation of COPD, infection can aggravate cough, increase sputum volume, and result in dyspnea [2, 3]. Infection control is a key measure in the treatment of acute exacerbation of elderly COPD. At present, antibiotics are generally used in clinical treatment, but the long-term application of antibiotics can cause drug-resistant strains, leading to flora imbalance and fungal infection [4].

According to the theory of traditional Chinese medicine, COPD belongs to “lung distension,” “asthmatic cough,” and phlegm blockages in lung collateral, accompanied by exogenous pathogenic qi, causing the stasis of heat-phlegm [4]. Xiyanping is a traditional Chinese medicine injection extracted and refined from Andrographis paniculata with antibacterial, antiviral, and other pharmacological effects, and it is widely used in infectious diseases such as bronchitis, tonsillitis, and bacterial diseases [5]. However, the studies on the efficacy of Xiyanping in COPD were few. The study is aimed at observing the influence of Xiyanping in elderly patients with COPD and its effect on the expression of GDF-15 and HIF-1*α* in serum. The report is as follows.

### 1.1. Core Tips

In this study, we found that Xiyanping could improve the pulmonary function of elderly patients with acute exacerbation of COPD, reduce the response of airway hyperreactivity, and promote the excretion of sputum, which might be related to the regulation of GDF-15 and HIF-1*α*-related factors.

## 2. Data and Methods

### 2.1. General Information

This study has been approved by the ethics committee. Diagnostic criteria in line with the standard of Chronic Obstructive Pulmonary Disease Diagnosis and Treatment Guidelines (2013 revision) [6] include (1) patients with COPD clinical symptoms, (2) patients who have a contact history of risk factors (including environmental factors and host factors), (3) FEV1/FVC that achieved 60%–80% after using a bronchodilator, and (4) chest X-ray/CT examination that showed increased lung texture, increased chest diameter, and increased lung field transparency.

Acute exacerbation of COPD was in line with the standard of AECOPD Diagnosis and Treatment of Chinese Expert Consensus (2017 update) [7]: (1) continuous deterioration of respiratory symptoms and (2) it is necessary to change the drug treatment plan.

### 2.2. Case Selection

Inclusion criteria include (1) meeting the criteria for acute exacerbation of COPD, (2) ages from 60 to 85 years without gender restriction, (3) excluding the related symptoms caused by tuberculosis and bronchiectasis, (4) patients and their families who agreed to join this study, and (5) complete clinical data.

Exclusion criteria include (1) in situ or metastatic lung cancer; (2) with previous history of pulmonary resection; (3) patients with defects in immune function; (4) bedridden or mobility-impaired patients; (5) patients with severe heart, liver, or kidney dysfunction; and (6) mental diseases.

### 2.3. Collection of Cases

From August 2019 to December 2021, 86 elderly patients with acute exacerbation of COPD admitted to our hospital were confirmed with the inclusion and exclusion criteria and were selected as the research subjects. As the research objects, they were divided into the control group (*n* = 43) and the observation group (*n* = 43) randomly. After the statistical test, it was found that the general information of them was balanced.

### 2.4. Method

The control group was given conventional treatment, including oxygen therapy, ambroxol phlegm, *β*2 receptor agonist bronchodilator, inhaled corticosteroids anti-inflammatory, broad-spectrum antibiotics, and other comprehensive treatment.

Based on the control group, the observation group was treated with Xiyanping injection (produced by China Jiangxi Qingfeng Pharmaceutical Co., Ltd., specification: 5 mL: 125 mg, SEDA approval number Z20026249). A total of 250 mg Xiyanping was added into 0.9% sodium chloride injection 250 mL for intravenous drip, one time per day. The two groups were evaluated after 14 days of treatment.

### 2.5. Detection Method

Before and after treatment, 10 mL of fasting venous blood samples was taken from patients with an empty stomach and divided into two vacuum blood vessels. One was detected by the Shenzhen Mairui five classification blood cell analyzer to test the blood routine for recording the levels of white blood cell count (WBC) and neutrophil ratio (NEU). The other one was centrifuged within 1 hour after blood collection with the rotating speed of 3500 r/min for 10 minutes. The serum was taken to detect GDF-15, HIF-1*α*, CXCL12, TNF-*α*, IL-8, and TGF-*β* by ELISA. The kits were all products of Shanghai Enzyme-Linked Biotechnology Co., Ltd., and the instrument was the Shenzhen Mairui RT-96A microplate reader.

Before and after treatment, CHEST GRAPHHI-10 Jester pulmonary function instrument was used to detect forced expiratory volume in the first second (FEV1) and forced vital capacity (FVC) and calculate FEV1/FVC in them. The BUXCO FinePointe RC lung compliance measurement system was used to detect airway resistance and lung compliance during exhalation and inspiration of airway hyperreactivity-related indexes in two groups.

### 2.6. Scoring Standard

*Chronic obstructive pulmonary assessment test (CAT) score [* 8 *]*: the evaluation is mainly aimed at the influence of patients' health and daily life with a total of eight items for the range from 0 to 40. The high or low score indicated that the influence of disease on health and daily life was large or small.

*Borg score [* 9 *]:* the degree of dyspnea was mainly evaluated, including blood oxygen saturation, heart rate, blood pressure, and respiratory frequency from the range of 0 to 10. The scores indicated the degree of dyspnea.

### 2.7. Statistical Method

Professional SPSS19.0 software was used for data processing; GDF-15, HIF-1*α*, lung function indicators, and other data which were in accordance with normal distribution should be described by $\bar{\chi }\pm s$; the *t*-test was used for comparison, count data was described by *n* (%), and the *χ*^2^ test was used for comparison, with statistical significance (*P* < 0.05).

## 3. Results

### 3.1. Differences in General Data between Two Groups

The process of the disease, the severity of illness, complications and smoking, age, and other general information were compared between the two groups, and there was no statistical difference (*P* > 0.05) (see Table 1).

### 3.2. Comparison of Sputum Excretion between Two Groups

There was nothing different in sputum excretion between them before treatment. On the 3rd and 7th days after being treated, the sputum excretion in them was higher than before, but on the 3rd day of treatment, the sputum excretion in the observation group was higher than that in the control group, while on the 7th day of treatment, the sputum excretion was lower than that in the control group with a statistically significant difference (*P* < 0.05) (see Table 2 and Figure 1).

### 3.3. Difference in Serum-Related Factors such as GDF-15 and HIF-1*α* between Two Groups

There was no difference in serum-related factors such as GDF-15 and HIF-1*α* between them before treatment. After treatment, GDF-15, HIF-1*α*, CXCL12, TNF-*α*, IL-8, and TGF-*β* in them were significantly lower than before, and the values in the observation group were significantly lower than those in the control group with a statistically significant difference (*P* < 0.05) (see Table 3).

### 3.4. Difference in Blood Routine Indexes between Two Groups

There was nothing different in blood routine indexes between them before treatment. After treatment, WBC and NEU in them were significantly lower than before, and values in the observation group were significantly lower than those in the control group (see Table 4).

### 3.5. Difference in Pulmonary Function Indexes between Two Groups

There was nothing different in pulmonary function indexes between them before treatment. After treatment, FEV1, FVC, and FEV1/FVC in them were significantly higher than before, and the values in the observation group were significantly higher than those in the control group with statistically significant differences (*P* < 0.05) (see Table 5).

### 3.6. Differences in Airway Hyperreactivity Indicators between the Two Groups

There was nothing different in the related indexes of airway hyperreactivity between them before treatment. After being treated, airway resistance and lung compliance of them at exhalation and inspiration were significantly lower than before, and the values in the observation group were significantly lower than those in the control group with a statistically significant difference (*P* < 0.05) (see Table 6).

### 3.7. Differences in CAT and Borg Scores between the Two Groups

There was nothing different in the CAT score and Borg score between them before treatment. After being treated, the CAT score and Borg score of them were significantly lower than before, and the value of the observation group was significantly lower than that of the control group with a statistically significant difference (*P* < 0.05) (see Table 7).

### 3.8. Differences in Duration of Antibiotic Use, Hospital Stays, and Adverse Reactions between the Two Groups

The duration of antibiotic use and hospital stays in the observation group were significantly shorter than those of the control group, while compared with the control group, there were no significant differences in the incidence of adverse reactions (*P* > 0.05) (see Table 8).

## 4. Discussion

An epidemiological survey shows that COPD ranks the sixth leading reason for death among the world's population and ranks 3rd among the causes of death from diseases in China. At present, there are about 100 million COPD patients in China, including about 30 million patients over 60 years old [10]. When they suffered from cold, infection, and inhalation of harmful gases, the symptoms would aggravate. In severe cases, respiratory failure and even death can occur [11]. At present, the routine treatment of western medicine for acute exacerbation of COPD can alleviate the clinical symptoms to some extent. However, the drug resistance of antibiotics makes the lower respiratory tract infection of a considerable number of patients unable to be effectively controlled; thus, it is difficult to achieve the ideal therapeutic effect [12].

According to the theory of traditional Chinese medicine, pathogenic qi which causes diseases invades the lung. The improper treatment leads to retention of pathogenic qi, and accumulation of phlegm and blood stasis damages healthy qi. Once the body is attacked by pathogenic qi, the sputum and blood stasis in the body will be invoked to aggravate cough and asthma. The therapeutic doctrine is heat-clearing and detoxifying, resolving phlegm, and relieving cough [13]. Xiyanping is a traditional Chinese medicine injection, and its active component is andrographolide sulfonate which was prepared by sulfonation of the extract from Andrographis paniculata leaves. The in vitro antibacterial experiments showed that it had obvious inhibitory effects on adenovirus, influenza virus, respiratory syncytial virus, and pathogenic microorganisms such as Staphylococcus aureus, Streptococcus, pneumococcal bacteria, and Escherichia coli. It is currently widely used in the treatment of respiratory and intestinal infectious diseases [14, 15].

In this study, it was found that the sputum excretion of the patients treated with Xiyanping adjuvant therapy was higher than that of the patients with conventional treatment 3 days later, while on the 7th day of treatment, the sputum excretion was lower than that in the control group. The CAT score and Borg score were lower than those of conventional treatment, and the duration of antibiotic use and hospital stays in the observation group were significantly shorter than those of the control group, while the incidence of adverse reactions in the two groups was similar. These results suggest that Xiyanping can not only better promote sputum excretion in elderly patients with acute exacerbation of COPD, reduce the symptom of dyspnea, accelerate the recovery process, and decrease the application of antibiotics but also not increase the risk of adverse reactions. Pulmonary function and airway responsiveness are clinical indicators for judging the severity and prognosis of COPD. In this study, it was found that FEV1, FVC, and FEV1/FVC of patients with Xiyanping adjuvant therapy after treatment were higher than those with conventional therapy, and their airway resistance and lung compliance during exhalation and inspiration were lower than those of patients with conventional therapy, suggesting that Xiyanping was conducive to improve lung function and reduce airway hyperreactivity in elderly patients with acute exacerbation of COPD. By introducing hydrophilic groups into the structure of andrographolide to enhance its antibacterial activity, Xiyanping prevents the proliferation and replication of viruses and bacteria by preventing protein from wrapping DNA fragments of pathogenic microorganisms and inhibits prostaglandin synthesis, protects lysosome membrane, reduces capillary permeability, and improves cellular immune function [16, 17]. In addition, Xiyanping also has an antagonistic effect on endotoxin. It can block LPS-mediated systemic inflammatory response and produce a good synergistic effect when combined with antibiotics [18, 19]. The lung ventilation function can be improved and airway hyperreactivity can be reduced when infection and inflammation are effectively controlled [20].

Local and systemic inflammatory response is an important pathological change in patients with acute exacerbation of COPD. WBC and NEU are immune cells of the body, which are highly expressed after infection and play their own anti-infection role [20–22]. GDF-15 is a stress response protein, which is mostly secreted by macrophages and adipocytes after activation to participate in physiological and pathological processes such as growing development and inflammatory reactions [23–25]. HIF-1*α* is a transcription factor regulating cells under hypoxic conditions, which can activate downstream inflammatory pathways and aggravate inflammatory injury of the respiratory tract [26]. CXCL12 is a member of the chemokine protein family, which forms a complex with the receptor and participates in the inflammatory response process [27, 28]. TNF-*α* is a proinflammatory factor synthesized by activated mononuclear macrophages, which can not only cause direct inflammatory injury in lung tissue but also promote the synthesis of other proinflammatory factors, such as IL-8, resulting in worsening tissue damage [29–31]. TGF-*β* can regulate cell growth and differentiation, inhibit immune cell differentiation and proliferation, and promote fibroblasts to release proinflammatory factors such as IL-6 [32–34]. In the study, it was found that the level of inflammatory indexes in the patients treated with Xiyanping adjuvant therapy was significantly lower than that in the patients treated with conventional therapy, suggesting that Xiyanping could regulate GDF-15 and HIF-1*α* to other inflammatory-related factors and reduce the inflammatory response of the body, which was one of the important mechanisms in the treatment of acute exacerbation of COPD in the elderly by detecting the above inflammatory indexes.

There were some limitations of this study. The sample size was limited. And this study was conducted in only one hospital. Thus, the results need to be confirmed by a multicenter randomized controlled study with a large cohort.

In summary, Xiyanping could improve the pulmonary function of elderly patients with acute exacerbation of COPD, reduce the response of airway hyperreactivity, and promote the excretion of sputum.

## Figures and Tables

**Figure 1:** Comparison of sputum excretion between the two groups. Before therapy, they were similar in the two groups. On the 3rd day after treatment, the sputum excretion of the observation group was higher than that of the control group. On the 7th day after treatment, the sputum excretion of the observation group was lower than that of the control group.

**Table 1:** Differences in general information between the two groups.

Normal information	Control group (*n* = 43)	Observation group (*n* = 43)	*χ* ^2^ or *t*	*P*
Gender (*n* (%))			0.191	0.662
Male	24 (55.81)	26 (60.47)		
Female	19 (44.19)	17 (39.53)		
Age ($\bar{\chi }\pm s$)	68.96 ± 5.77	69.21 ± 5.23	0.211	0.834
BMI ($\bar{\chi }\pm s$) (kg/m^2^)	22.33 ± 2.16	21.98 ± 2.24	0.738	0.463
Severity of illness (*n* (%))			0.508	0.476
Moderate	32 (74.42)	29 (67.44)		
Severe	11 (25.58)	14 (32.56)		
COPD course of disease ($\bar{\chi }\pm s$) (year)	10.25 ± 3.11	10.08 ± 2.98	0.259	0.796
Smoking status (*n* (%))			0.426	0.808
None	24 (55.81)	21 (48.84)		
Quit smoking	8 (18.60)	9 (20.93)		
Smoking	11 (25.58)	13 (30.23)		
Concomitant disease (*n* (%))				
Hypertension	17 (39.53)	20 (46.51)	0.427	0.514
Diabetes	15 (34.88)	12 (27.91)	0.486	0.486
Coronary heart disease	12 (27.91)	16 (37.21)	0.847	0.357
Hyperlipidemia	18 (41.86)	17 (39.53)	0.048	0.826

**Table 2:** Comparison of expectoration between the two groups.

Group	*n*	Expectoration ($\bar{\chi }\pm s$) (mL)		
		Before therapy	Treatment 3 d	Treatment 7 d
Control group	43	28.65 ± 7.46	74.11 ± 12.41^∗^	86.32 ± 14.79^∗^
Observation group	43	27.91 ± 8.03	105.45 ± 15.63^∗^	34.55 ± 9.45^∗^
*t*		0.443	10.297	19.342
*P*		0.659	<0.001	<0.001

Compared with before treatment, ^∗^*P* < 0.05.

**Table 3:** Differences in serum-related factors such as GDF-15 and HIF-1*α* between them ($\bar{\chi }\pm s$).

Group	*n*	GDF-15 (*μ*g/L)		HIF-1*α* (ng/L)		CXCL12 (ng/L)	
		Before	After	Before	After	Before	After
Control group	43	2.85 ± 0.49	1.65 ± 0.38^∗^	30.58 ± 8.99	18.11 ± 6.43^∗^	314.52 ± 74.96	274.63 ± 54.14^∗^
Observation group	43	2.79 ± 0.55	1.21 ± 0.27^∗^	29.97 ± 9.07	11.42 ± 4.45^∗^	305.88 ± 79.11	213.52 ± 43.63^∗^
*t*		0.534	6.190	0.313	5.610	0.520	5.763
*P*		0.595	<0.001	0.755	<0.001	0.605	<0.001
Group	*n*	TNF-*α* (*μ*g/L)		IL-8 (*μ*g/L)		TGF-*β* (ng/mL)	
		Before	After	Before	After	Before	After
Control group	43	4.15 ± 0.58	3.21 ± 0.52^∗^	104.52 ± 27.65	38.56 ± 12.41^∗^	71.56 ± 24.41	52.05 ± 17.79^∗^
Observation group	43	4.06 ± 0.61	2.55 ± 0.43^∗^	101.78 ± 31.64	21.35 ± 8.25^∗^	68.96 ± 25.56	41.31 ± 14.66^∗^
*t*		0.701	6.414	0.428	7.573	0.482	3.055
*P*		0.485	<0.001	0.670	<0.001	0.631	0.003

Compared with before treatment, ^∗^*P* < 0.05.

**Table 4:** Differences in blood routine indexes between the two groups ($\bar{\chi }\pm s$).

Group	*n*	WBC (×10^9^/L)		NEU (%)	
		Before	After	Before	After
Control group	43	12.23 ± 2.89	8.87 ± 1.97^∗^	87.45 ± 8.63	76.64 ± 6.49^∗^
Observation group	43	12.31 ± 2.57	7.18 ± 1.54^∗^	85.97 ± 8.44	69.85 ± 5.14^∗^
*t*		0.136	4.432	0.804	5.378
*P*		0.892	<0.001	0.424	<0.001

Compared with before treatment, ^∗^*P* < 0.05.

**Table 5:** Differences in pulmonary function indexes between the two groups ($\bar{\chi }\pm s$).

Group	*n*	FEV1 (L)		FVC (L)		FEV1/FVC (%)	
		Before	After	Before	After	Before	After
Control group	43	1.21 ± 0.49	1.68 ± 0.52^∗^	2.04 ± 0.59	2.46 ± 0.61^∗^	53.25 ± 8.47	66.56 ± 7.56^∗^
Observation group	43	1.23 ± 0.43	2.19 ± 0.61^∗^	2.11 ± 0.58	2.89 ± 0.64^∗^	55.04 ± 8.29	75.48 ± 6.04^∗^
*t*		0.201	4.172	0.555	3.189	0.990	6.045
*P*		0.841	<0.001	0.580	0.002	0.325	<0.001

Compared with before treatment, ^∗^*P* < 0.05.

**Table 6:** Differences in airway hyperreactivity indicators between the two groups ($\bar{\chi }\pm s$).

Group	*n*	Airway resistance during exhalation (cm H_2_O/(L·s))		Airway resistance during inspiration (cm H_2_O/(L·s))		Lung compliance (mL/cm H_2_O)	
		Before	After	Before	After	Before	After
Control group	43	1.87 ± 0.74	1.42 ± 0.51^∗^	1.81 ± 0.89	1.54 ± 0.41^∗^	174.25 ± 45.36	135.26 ± 31.05^∗^
Observation group	43	1.89 ± 0.69	1.21 ± 0.43^∗^	1.86 ± 0.82	1.28 ± 0.37^∗^	169.85 ± 48.14	108.57 ± 24.96^∗^
*t*		0.130	2.064	0.271	3.087	0.436	4.393
*P*		0.897	0.042	0.787	0.003	0.664	<0.001

Compared with before treatment, ^∗^*P* < 0.05.

**Table 7:** Differences in CAT scores and Borg scores between the two groups (($\bar{\chi }\pm s$), fraction).

Group	*n*	CAT score		Borg score	
		Before	After	Before	After
Control group	43	17.05 ± 5.94	11.89 ± 2.16^∗^	8.87 ± 2.07	6.13 ± 1.88^∗^
Observation group	43	16.53 ± 6.17	9.23 ± 2.07^∗^	8.95 ± 2.13	4.57 ± 1.29^∗^
*t*		0.398	5.830	0.177	4.487
*P*		0.692	<0.001	0.860	<0.001

Compared with before treatment, ^∗^*P* < 0.05.

**Table 8:** Differences in duration of antibiotic use, length of stay, and adverse reactions between the two groups.

Group	*n*	Antibiotic use time ($\bar{\chi }\pm s$) (d)	Hospital stay ($\bar{\chi }\pm s$) (d)	Adverse reactions (*n* (%))			
				Rash	Diarrhea	Irritable	Total
Control group	43	8.47 ± 1.89	13.07 ± 2.57	1 (2.33)	2 (4.65)	0 (0.00)	3 (6.98)
Observation group	43	6.35 ± 1.41	9.84 ± 1.93	2 (4.65)	1 (2.33)	1 (2.33)	4 (9.30)
*t* or *χ*^2^		5.896	6.590				0.156
*P*		<0.001	<0.001				0.693

## Data Availability

The datasets used and analyzed during the current study are available from the corresponding author upon reasonable request.
